# Computed Tomography Images under Artificial Intelligence Algorithms on the Treatment Evaluation of Intracerebral Hemorrhage with Minimally Invasive Aspiration

This article has been retracted.

**DOI:** 10.1155/2022/6204089

**Published:** 2022-04-22

**Authors:** Junfeng Sun, Xiaojun Zheng, Qiang Gao, Xiaofeng Wang, Yu Qiao, Jialong Li

**Affiliations:** ^1^Department of Neurosurgery, Baoji People's Hospital, Baoji, 721000 Shaanxi, China; ^2^Department of Neurology, Baoji People's Hospital, Baoji, 721000 Shaanxi, China; ^3^Department of Neurosurgery, Third Hospital of Baoji City, Baoji, 721000 Shaanxi, China

## Abstract

The aim of this study was to investigate the therapeutic effect of minimally invasive aspiration on intracerebral hemorrhage (ICH) and the value of artificial intelligence algorithm combined with computed tomography (CT) image evaluation. Ninety-two patients with intracerebral hemorrhage were divided into experimental group (46 cases, minimally invasive aspiration therapy) and control group (46 cases, traditional craniotomy therapy) according to different treatment methods, and CT image scanning was performed. In addition, a CT image segmentation model of intracerebral hemorrhage based on improved fuzzy C-means clustering algorithm (n-FCM) was proposed to process the CT images of the patients. The results showed that the Dice coefficient of n-FCM algorithm after the addition of salt and pepper noise was 0.89, which was higher than that of traditional algorithm; the average operation time of experimental group was 58.93 ± 5.33 min, which was significantly lower than that of control group (90.21 ± 16.24 min) (*P* < 0.05); the overall response rate of experimental group was 93.48%, which was significantly higher than that of control group (76.09%) (*P* < 0.05); one month after operation, the *National Institutes of Health Stroke Scale* (NIHSS) score of experimental group was 3.89 ± 1.95 points, and the *Scandinavian Stroke Scale* (SSS) score was 10.67 ± 1.76 points, which was significantly lower than that of control group (*P* < 0.05); the incidence rate of complications in experimental group was significantly lower than that of control group (*P* < 0.05). It showed that the n-FCM algorithm was superior to the traditional algorithm in CT image processing, with the advantages of good denoising effect and less running time. Minimally invasive aspiration treatment had the advantages of operation time, convenient operation, and less damage to patients, which was beneficial to postoperative recovery and prognosis of patients.

## 1. Introduction

Intracerebral hemorrhage (ICH) is a common disease. It is generally divided into nontraumatic hemorrhage and traumatic hemorrhage according to the cause of the disease, and both have a high mortality and disability rate, causing serious health hazards and economic burdens for patients and their families [1–3]. Effective removal of hematoma is the key to the treatment of ICH. The removal of hematoma is conducive to reducing the patient's intracranial pressure, thereby improving cerebral perfusion and achieving the treatment [4, 5]. At present, the common methods for clinical treatment of ICH include conservative medical treatment and craniotomy debridement [6]. However, according to clinical studies, neither of the above two methods can improve the prognosis of patients [7]. Among them, craniotomy is more traumatic and easy to damage the blood vessels around the hematoma and often has complications such as intracranial infection and is affected by the patient's bleeding site and bleeding volume, and its clinical application is severely limited [8, 9]. With the rapid development of medical technology, minimally invasive aspiration drainage is gradually being carried out clinically. This technology has the characteristics of accurate positioning, convenient operation, and small surgical trauma. It has become one of the commonly used methods for the treatment of ICH [10]. Minimally invasive aspiration drainage is divided into hard channel minimally invasive aspiration drainage and soft channel minimally invasive removal. Clinically, different surgical procedures are used according to the specific conditions of the patient and have different prognosis.

Computed tomography (CT) is an important imaging examination for ICH patients, and its imaging results are important indicators for analyzing intracranial hemorrhage [11]. Manual segmentation and automatic segmentation are commonly used in clinical practice to achieve quantitative segmentation of intracranial hematoma. Between them, manual segmentation has poor repeatability and is time-consuming, and its segmentation accuracy needs to be studied and is affected by the experience and level of clinicians; there are situations where there are different segmentation results in the same case [12, 13]. On the other hand, it is difficult for even experienced doctors to completely segment the specific situation of intracranial hematoma due to the problems of complicated shapes and unclear borders in CT imaging of ICH patients [14]. With the continuous improvement and development of artificial intelligence algorithms, it has been widely used in the field of medical imaging. Among them, the fuzzy C-means (FCM) algorithm has shown superiority in the field of image segmentation. Kavitha et al. [15] proposed a region-based FCM for segmentation of lung cancer regions and classification based on support vector machine (SVM) to diagnose cancer stages. The comparative experiments showed that the designed model had obvious advantages in improving diagnosis accuracy and reducing error rate.

In summary, ICH has a high rate of death and disability, causing serious psychological pressure and financial burden to patients and their families. Minimally invasive aspiration drainage has the advantages of convenient operation and small surgical wounds in the treatment of ICH. However, the segmentation results are affected by CT imaging. Therefore, a CT image model of intracranial hemorrhage based on the improved FCM algorithm was proposed and applied to evaluate the clinical application effect of minimally invasive aspiration drainage, and it was expected to provide a number of evidences for clinical treatment strategies for ICH patients.

## 2. Research Materials and Methods

### 2.1. Research Objects and Their Groups

Ninety-two patients who were treated at the hospital from April 2018 to July 2020 were selected as the research objects. According to the different treatment methods, they were divided into an experimental group and a control group, with 46 patients in each group. The patients in the control group underwent traditional craniotomy debridement, and patients in the experimental group underwent minimally invasive aspiration drainage treatment. The general clinical data of patients were collected, and CT examinations were performed on all patients. This study had been approved by the ethics committee of hospital, and the patients and their families had understood the experiment and signed the informed consent forms.

Inclusion criteria are as follows: all patients underwent CT examination, which met the ICH diagnostic criteria, and the bleeding site was clarified; the general clinical data of the patients were complete; the patients were 18 to 73 years old; all patients had indications for surgery; and pregnancy. Exclusion criteria are as follows: patients with poor compliance; patients with intracranial hemorrhage caused by trauma; patients with surgical contraindications; patients combined with malignant tumor; and patients with major surgery recently.

### 2.2. Treatment Methods

#### 2.2.1. Traditional Craniotomy and Debridement

The patients were scanned by CT. The scanning parameters were set as follows: tube voltage was 120 kV, tube current was 200 mA, pitch was 1.0, layer thickness was 1.0 mm, and matrix was 512 × 512. After the scan, 2 experienced clinical imaging doctors manually segmented it to confirm the size and location of the lesion. It should routinely drape and disinfect after general anesthesia, cut the skin tissue to expose the skull, and use a skull electric drill to drill holes. Taking the hematoma site as the central opening about 5 cm bone window, the heart milled the bone flap along the skull hole to expose the dura mater. After the extradural hematoma was removed, it should cut the dura mater to expose the hematoma site and surrounding area directly to the hematoma cavity. A suction device and bipolar coagulation were adopted to remove the hematoma and the surrounding necrotic brain tissue. After the hematoma was removed, the issue was rinsed with normal saline. Finally, after the drainage tube was placed successfully, the dura mater, surrounding tissues, and scalp that were cut during the operation should be sutured.

#### 2.2.2. Minimally Invasive Aspiration Drainage

After CT scan, it should confirm the bleeding site and make a puncture plan. Routine drapes were disinfected with lidocaine (2 mL: 4 mg) with local anesthesia. An electric drill was adopted to penetrate the scalp and subcutaneous tissue to pierce the YL-1 puncture needle under the skull at the lesion site, avoiding important blood vessels and tissues. After the electric drill was removed, it should advance the puncture needle into the lesion, and pull out the needle core link aspirator to slowly suck the hemorrhage. Then, the tissue was rinsed with normal saline to anhydrous water, and the drainage tube was connected and wrapped with a sterile dressing. After the operation, 20,000 U of urokinase was injected through the drainage tube, and the tube was clamped for 2 hours before the drainage was opened.

### 2.3. FCM Algorithm and Its Optimization

The FCM algorithm was improved based on the K-means clustering algorithm. In the K-means clustering algorithm, *X* objects were divided into *K* categories according to certain attributes. Therefore, in medical imaging, each pixel of an image corresponded to a cluster. In FCM, the membership function *α*_*xy*_ was used to indicate that the first object belongs to the *x*-th cluster, and the equation was expressed as follows.

(1) $$\begin{array}{c} Q=\Sigma \begin{array}{c} Y\\ y=1 \end{array}\Sigma \begin{array}{c} W\\ x=1 \end{array}\alpha_{xy}^{1}{\left\|r_{y}-q_{x}\right\|}^{2}. \end{array}$$

*m* was adopted to represent the value of the fuzzy parameter. When *m* = 2, it satisfied the below equation.

(2) $$\begin{array}{c} T\in \left\{\alpha_{ir}\in \left[0,1\right]\right|\Sigma_{i=1}^{W}\alpha_{ir}=1,\forall k\text{ and }0<\Sigma \begin{array}{c} Y\\ k=1 \end{array}\alpha_{ir}<Y,\forall i. \end{array}$$

The objective function was minimized: pixels would be assigned a high degree of membership when they were close to the cluster centroid. The degree of membership depended on the distance of each individual cluster center. In FCM, *α*_*xy*_ and centroid *p*_*r*_ were expressed by

(3) $$\begin{array}{c} \alpha_{xy}=\frac{\alpha_{xy}^{1}{\left\|i_{y}-q_{x}\right\|}^{-2/l-1}}{\Sigma_{k=1}^{W}{\left\|i_{y}-q_{k}\right\|}^{-2/l-1}}, \end{array}$$

(4) $$\begin{array}{c} p_{r}=\frac{\Sigma_{y=1}^{W}\alpha_{xy}^{1}r_{y}}{\Sigma_{y=1}^{W}\alpha_{xy}^{1}}. \end{array}$$

The FCM algorithm showed good segmentation performance, but its segmentation performance was greatly reduced in noisy images, and it was very sensitive to false negatives. The main reason was that the FCM algorithm used Euclidean distance, which had poor robustness and was poorly sensitive to spatial information in the image. Therefore, it was considered to improve FCM from two aspects of robustness and spatial information. The relationship among neighboring pixels in spatial information was a very important factor. In most edge detection algorithms, the relationship between neighboring pixels had been used to achieve excellent image segmentation. The improved algorithm redefined the objective function, added space constraints in it, and used space instead of the membership function in the original FCM algorithm. The equation was as follows.

(5) $$\begin{array}{c} Q_{x}=\Sigma \begin{array}{c} W\\ i=1 \end{array}\Sigma \begin{array}{c} Y\\ k=1 \end{array}\alpha_{ik}^{x}{\left\|m_{k}-q_{i}\right\|}^{2}+\mu \Sigma \begin{array}{c} W\\ i=1 \end{array}\Sigma \begin{array}{c} Y\\ k=1 \end{array}\mu_{ik}^{x}{\left\|{\overset{-}{m}}_{k}-q_{i}\right\|}^{2},\\ f_{ig}=\Sigma_{k\in SD\left(mg\right)}\alpha_{ik},\alpha_{ik}^{l}=\frac{\alpha_{ik}f_{ig}}{\Sigma_{k=1}^{W}\alpha_{ik}f_{ig}}. \end{array}$$

In the above equation, *f*_*ig*_ represented the possibility that the *g*-th pixel belongs to the *i*-th cluster, and the centroid of the cluster can be updated according to equation (4), which could be expressed as

(6) $$\begin{array}{c} \left\|Q_{new}-Q_{old}\right\|<\varepsilon \;Q=\left[q_{1},q_{2},\cdots ,q_{w}\right]. \end{array}$$

The improved FCM model was set as n-FCM. *A* was adopted to represent the area manually segmented by the expert, and *B* represented the area automatically segmented by the algorithm. The value of the Dice coefficient ranged from 0 to 1. The larger the value, the better the segmentation effect of the algorithm; the smaller the value, the poorer the segmentation effect of the algorithm or the segmentation error.

(7) $$\begin{array}{c} DC=\frac{2\left|A⋂B\right|}{\left|A\right|+\left|B\right|}. \end{array}$$

### 2.4. Observation Indicators

The observation indicators included patient's hospitalization time, operation time, and hematoma on the first day and one week after the operation. The *Scandinavian Stroke Scale* (SSS) [16] was used to evaluate the patient's neurocognitive function impairment; the lower the score, the better the neurocognitive function; the *National Institutes of Health Stroke Scale* (NIHSS) [17] was used to evaluate the patient's neurocognitive function recovery; the lower the score, the better the recovery of neurocognitive function. The efficacy evaluation criteria were given as follows. The treatment effect was significant: the clinical symptoms had basically disappeared, no additional surgical treatment was required, and the prognosis was good without complications. The treatment was effective: the patient's clinical symptoms were alleviated, and there were fewer postoperative complications. The treatment was ineffective: the patient's clinical symptoms had not been relieved, the patient needed another surgical treatment, and the postoperative complications were serious. Total effective rate = (effective + significant effect)/total number of cases × 100%.

### 2.5. Statistical Analysis

SPSS20 system was used for data analysis, measurement data was expressed as $\bar{x}\pm \text{s}$, and independent sample *t*-test analysis was used for comparison between groups. The repeated measurement data analysis of variance was used for multiple time periods, count data were expressed as percentages, and *χ*^2^ test was adopted. *P* < 0.05 indicated statistical significance.

## 3. Results

### 3.1. Algorithm Performance Analysis

In order to verify the segmentation performance of the improved algorithm, the S-FCM algorithm [18] was introduced, and the segmentation performance of the three algorithms was compared in a system environment with a 3.0 GHz memory of 2 GB. In addition, the salt and pepper noise was added. The results were shown in Figure 1. The Dice coefficient value of the FCM algorithm before adding noise was 0.79, and the S-FCM algorithm was 0.85, which were both smaller than the improved algorithm (0.97). After the salt and pepper noise was added, the Dice coefficient value of the n-FCM algorithm was 0.89, which was higher than that of the FCM and S-FCM algorithms.

The operation time and clustering times of the three algorithms after addition of salt and pepper noise were compared, and the results were shown in Figure 2. It can be observed that the S-FCM algorithm showed the least clustering times among the three algorithms. The clustering times of the FCM algorithm was similar to that of the n-FCM algorithm; the calculation time of the S-FCM algorithm was 32.15 seconds, the shortest calculation time of the FCM algorithm was 9.44 seconds, and the calculation time of the n-FCM algorithm was 11.34.

### 3.2. Comparison of Segmentation Results

The segmentation effect diagrams of the three algorithms were shown in Figure 3. Figure 3 showed the CT images of a patient with ICH. It can be observed that the shape of the hematoma was relatively irregular, and there was a low-density cerebral edema zone around the hematoma. It can be concluded from the segmentation results of the three algorithms that the traditional FCM algorithm segmentation edge was relatively fuzzy and presented an irregular edge. The segmentation result of S-FCM algorithm was slightly better than that of traditional FCM algorithm, and obvious segmentation contours can be observed. The segmentation result of the n-FCM algorithm was the clearest, and the segmentation contour edge was clearly visible.

In order to further verify the effect of the improved FCM algorithm on noise processing, the salt and pepper noise was added. The segmentation results of the three algorithms were shown in Figure 4. It can be observed that the addition of salt and pepper noise would affect the segmentation results of the three algorithms and additionally increased the calculation time of the algorithm. The results suggested that the n-FCM algorithm had a certain effect on noise processing. Compared with the traditional FCM algorithm and the S-FCM algorithm, the segmentation result of n-FCM algorithm was more accurate.

### 3.3. Statistics of General Clinical Data of Patients

The general clinical data statistics of the two groups of patients were shown in Table 1. In the experimental group, there were 19 males and 27 females; the average systolic blood pressure was 162.54 ± 19.22 mmHg, and the average diastolic blood pressure was 98.43 ± 17.03 mmHg; and the average age of the patients was 63.42 ± 5.21 years old. In addition, 31 cases were located in the basal ganglia and 15 cases were located under the cortex; and the average blood loss was 51.23 ± 7.21 mL. There was no statistically significant difference in the above clinical items between the experimental group and the control group (*P* > 0.05).

### 3.4. Comparison of Operation Time, Hospital Stay, and Hematoma Size before and after Surgery

The average operation time of patients in the experimental group was 58.93 ± 5.33 min, which was significantly shorter than that of the control group (90.21 ± 16.24 min, and the difference was statistically significant (*P* < 0.05). The average hospital stay of patients in the experimental group was 10.03 days, which was obviously lower than that of patients in the control group (16.31 days), and the difference was statistically significant (*P* < 0.05), as shown in Figure 5(a). The volume of hematoma in the experimental group was 21.44 ± 3.24 mL and 7.89 ± 2.45 mL at 1 day and 1 week after surgery, respectively; the volume of hematoma in the control group was 19.32 ± 4.26 mL and 7.24 ± 2.61 mL at 1 day and 1 week after surgery, respectively, showing statistically significant difference (*P* < 0.05), as shown in Figure 5(b).

### 3.5. Comparison of Treatment Effect between Two Groups of Patients

In the experimental group, there were 30 patients with significant treatment effect, 13 patients with effective treatment, and only 3 patients with ineffective treatment. In the control group, there were 12 patients with significant treatment effect, 23 patients with effective treatment, and 11 patients with ineffective treatment. The total effective rate of treatment in the experimental group was 93.48%, which was significantly higher than that in the control group (76.09%), and the difference was statistically significant (*P* < 0.05), as shown in Figure 6.

### 3.6. Comparison of Nerve Function between Two Groups of Patients before and after Surgery

The preoperative NIHSS of the experimental group and the control group were 8.45 ± 3.21 points and 8.31 ± 2.78 points, respectively, and the difference was not statistically significant (*P* > 0.05). One month after the surgery, the NIHSS score of the experimental group was 3.89 ± 1.95 points, which was much lower than that of the control group (4.95 ± 2.33 points), and the difference was statistically significant (*P* < 0.05), as shown in Figure 7(a). The preoperative SSS of the experimental group and the control group were 27.97 ± 5.32 points and 27.43 ± 4.86 points, respectively, and the difference was not statistically significant (*P* > 0.05). One month after surgery, the SSS score of the experimental group was 10.67 ± 1.76 points, which was obviously lower than that of the control group (16.98 ± 2.68 points), and the difference was statistically significant (*P* < 0.05), as shown in Figure 7(b).

### 3.7. The Occurrence of Postoperative Complications in the Two Groups of Patients

In the experimental group, the postoperative incidences of gastrointestinal hemorrhage, urinary tract infection, lung infection, intracranial rebleeding, and intracranial infection were 4.35%, 0%, 2.17%, 2.17%, and 4.35%, respectively, which were significantly lower than those in the control group. The difference was statistically significant (*P* < 0.05), as shown in Figure 8.

## 4. Discussion

The mortality rate of ICH is extremely high. Studies have reported that the mortality rate within 30 days is about 50%. Even if the patients are lucky enough to survive, most of them have difficulty returning to normal lives [19]. At present, the common clinical treatment methods are internal conservative treatment and surgical treatment. Minimally invasive surgery has been confirmed by most studies. It is a new method to improve prognosis and reduce deaths [20]. Gui et al. [21] analyzed the effects of neuroendoscopic minimally invasive surgery and small bone window craniotomy to remove hematoma. The results showed that neuroendoscopic surgery for the treatment of hypertension with smaller bone window craniotomy is more effective, safer, less bleeding, better prognosis, and better nerve function recovery. Therefore, an ICH CT image segmentation model based on the improved FCM algorithm was constructed and used in minimally invasive aspiration treatment of ICH. In addition, the segmentation performance of the traditional FCM algorithm, S-FCM algorithm, and n-FCM algorithm was compared. The results revealed that the n-FCM algorithm showed a good segmentation effect among the three algorithms, and the Dice coefficient value of the n-FCM algorithm was 0.89. Chen et al. [22] avoided the label image and supervision, directly realized the calculation of the loss function of the FCM algorithm in the image itself, and confirmed the effectiveness and stability of the algorithm.

According to different treatment methods, 92 patients with intracerebral hemorrhage were divided into experimental group (minimally invasive aspiration therapy) and control group (traditional craniotomy therapy). The surgery-related indicators of the two groups were compared firstly. The results showed that the average operation time of the experimental group was 58.93 ± 5.33 min, and the average hospital stay was 10.03 days, which were significantly lower than those of the control group (*P* < 0.05). This was similar to the findings of Minhas et al. [23]. Minimally invasive aspiration treatment is to use the convenience of puncture needle operation to perform cranial puncture at the hematoma site, which effectively avoids damage to the surrounding tissues of the bleeding site and can go directly to the lesion to clear the hematoma. The hematoma volume of patients in the experimental group was 21.44 ± 3.24 mL and 7.89 ± 2.45 mL at 1 day and 1 week after surgery, respectively; the hematoma volume of patients in the control group was 19.32 ± 4.26 mL and 7.24 ± 2.61 mL at 1 day and 1 week after surgery, respectively, showing statistically significant differences (*P* < 0.05). However, the difference between the experimental group and the control group was not significant. The postoperative neurological function of the two groups of patients was compared. The results showed that the NIHSS score and the SSS score of the experimental group were 3.89 ± 1.95 points and 10.67 ± 1.76 points in the experimental group one month after the surgery, which were significantly lower than those of the control group, and the difference was statistically significant (*P* < 0.05). Cavallo et al. [24] conducted a systematic review on the application of minimally invasive aspiration in ICH, and the results showed that minimally invasive technology is still in dispute in the treatment of ICH. However, many clinical studies have shown that minimally invasive treatment is associated with significantly improved results compared with conservative treatment and traditional surgical removal strategies.

30 patients in the experimental group had a significant treatment effect, and their total effective rate of treatment was 93.48%, which was significantly higher than that in the control group (76.09%), showing statistically significant difference (*P* < 0.05). Minimally invasive surgery for the treatment of ICH is not just minimally invasive aspiration. Ziai et al. [25] explored the application effect of minimally invasive surgery combined with alteplase in the treatment of ICH. Kellner et al. [26] explored the minimally invasive endoscopic assessment of long-term functional results after ICH removal, and it showed that this method may produce favorable long-term functional results. But no matter which method is used, postoperative complications are problems that need to be solved urgently. The incidences of postoperative gastrointestinal hemorrhage, pulmonary infection, intracranial rebleeding, and intracranial infection were 4.35%, 2.17%, 2.17%, and 4.35%, respectively. All these values were significantly lower than those in the control group, and there were statistically significant differences (*P* < 0.05). The main reasons for complications are long-term hypertension, severe atherosclerosis, and damage of operation to other tiny nerves and blood vessels, which further increases the risk of intracranial hemorrhage after surgery [27]. On the other hand, patients need to stay in bed strictly after surgery, and they have weak cough and sputum due to the wound, which also increases the risk of lung infection [28]. Furthermore, patients have strict dietary taboos due to nerve function and body damage, which can easily cause gastrointestinal bleeding [29].

## 5. Conclusion

It was to analyze the application effect of minimally invasive aspiration in the treatment of ICH using CT images based on intelligent algorithms. A CT ICH image segmentation model based on the improved FCM algorithm was proposed, and the segmentation performance of which was compared with that of the traditional FCM algorithm and the S-FCM algorithm. 92 patients with ICH were selected as the research objects and divided into a traditional craniotomy control group and a minimally invasive aspiration treatment experimental group according to the treatment method. The postoperative treatment effect, neurological cognitive function, and postoperative complications of the two groups of patients were compared and analyzed. The results showed that minimally invasive aspiration treatment had the advantages of operation time, short hospitalization time, convenient operation, and less damage to the patient. Therefore, it was conducive to postoperative recovery and prognosis. However, there were certain limitations. The study follow-up time was short, and the long-term effects of the experimental group cannot be observed. In the future, more in-depth performance analysis of the improved FCM model will be carried out, and the data of patients with larger sample size will be collected to further explore the clinical treatment of patients with intracerebral hemorrhage. In general, it provided data support for the selection of treatment methods for ICH patients.

## Figures and Tables

**Figure 1:** Comparison on algorithm segmentation performance before and after the addition of noise. (a) The comparison of original CT image Dice before the salt and pepper noise was added and (b) the comparison of CT image Dice after the salt and pepper noise was added.

**Figure 2:** Comparison of operation time and clustering times. (a) The comparison of the number of clusters and (b) the comparison of the operation time.

**Figure 3:** Comparison of the segmentation results of the three algorithms. (a) showed the image to be segmented; (b) and (c) were the segmentation results of the traditional FCM algorithm; (d) and (e) were the segmentation results of the S-FCM algorithm; and (f) and (g) were the n-FCM segmentation results.

**Figure 4:** Comparison of the segmentation results of the three algorithms after addition of salt and pepper noise. (a) showed the image to be segmented; (b) and (c) were the segmentation results of the traditional FCM algorithm; (d) and (e) were the segmentation results of the S-FCM algorithm; and (f) and (g) were the n-FCM segmentation results.

**Figure 5:** Comparison of operation time, hospitalization time, and preoperative and postoperative hematoma size between the two groups. (a) showed the comparison between operation time and hospitalization time; (b) showed the comparison of hematoma size before and after the operation. ∗ indicated that the difference was statistically significant compared to the experimental group (*P* < 0.05); # indicated that the difference was statistically significant compared to preoperation (*P* < 0.05).

**Figure 6:** Comparison of treatment effects between the two groups of patients. (a) showed the statistics of the number of people; (b) showed the comparison of effective rates. ∗ meant that the difference was statistically significant compared to the experimental group (*P* < 0.05).

**Figure 7:** Comparison of NIHSS and SSS scores between the two groups of patients before and after surgery. (a) showed the comparison of the NIHSS score; (b) showed the comparison of the SSS score. ∗ meant that the difference was statistically significant compared to the experimental group (*P* < 0.05).

**Figure 8:** Comparison of the incidence of postoperative complications between the two groups of patients. (a)~(e) showed the incidence of gastrointestinal bleeding, urinary tract infection, lung infection, intracranial rebleeding, and intracranial infection, respectively. ∗ meant that the difference was statistically significant compared to the experimental group (*P* < 0.05).

**Table 1:** Comparison of general clinical data of patients.

Item	Experimental group (*n* = 46)	Control group (*n* = 46)
Gender (*n*)		
Males	19	20
Females	27	26
Blood pressure (mmHg)		
Systolic	162.54 ± 19.22	161.39 ± 18.92
Diastolic	98.43 ± 17.03	96.97 ± 18.14
Age (years old)	63.42 ± 5.21	61.78 ± 4.95
Bleeding site (*n*)		
Basal ganglia	31	34
Under the cortex	15	12
Preoperative blood loss (mL)	51.23 ± 7.21	50.21 ± 6.58

## Data Availability

The data used to support the findings of this study are available from the corresponding author upon request.
